The article "Clinical Significance of Detection of Peripheral Blood VASP Level in Lung Cancer Patients" was retracted in 2023. Reasons: unreliable results or conclusions; lack of ethics approval or compliance; concerns about the data; concerns about the peer review.

# Clinical Significance of Detection of Peripheral Blood VASP Level in Lung Cancer Patients

**DOI:** 10.1155/2022/1703339

**Published:** 2022-07-31

**Authors:** Jin Ma, Shumin Zhu, Zhiqing Chen, Xinyuan Li, Yafei Mao, Xin Tian, Li Zhao, Yanming Li, Baoqin Li, Yulan Geng

**Affiliations:** ^1^Laboratory, The Third Hospital of Hebei Medical University, Shijiazhuang 050051, Hebei Province, China; ^2^Laboratory, The First Hospital of Hebei Medical University, Shijiazhuang 050030, Hebei Province, China

## Abstract

This paper explores the relationship between the clinical value of vasodilator-stimulated phosphoprotein (VASP) in lung cancer tissue and its diagnosis and severity. Totally 100 patients who were clinically diagnosed with lung cancer from January 2018 to December 2020 were enrolled in our study. They were assigned into two groups according to the presence of lymph node metastasis. The VASP levels were measured by flow cytometry. The correlation between the expression of VASP in tumor tissue and the clinical characteristics and prognosis in patients was analyzed. The diagnostic efficacy of plasma VASP with squamous cell carcinoma antigen (SCC), neuron-specific enolase (NSE), cytokeratin-19 fragment (CYFRA21-1), prosecretin-releasing peptide (proGRP), and lung cancer was analyzed. The results were compared with APACHE III score to evaluate the accuracy of VASP in determining the severity of patients. This paper finds that the value of VASP in the non-lymph node metastasis group was significantly higher than that in the healthy control group, and the VASP level in the lymph node metastasis group was significantly higher than that in the non-lymph node metastasis group and the healthy control group (all *p* values <0.05). The APACHE III score of the lymph node metastasis group was higher than that of the non-lymph node metastasis group (*p* value <0.05). The diagnostic efficacy of VASP is similar to that of SCC, NSE, CYFRA21-1, and proGRP. The plasma VASP value was statistically different in the survival group and the death group, with higher level observed in the death group compared to survival group (all *p* values <0.05). The value of plasma VASP alone and acute physiology and chronic health evaluations III (APACHE III) score for lung cancer mortality was similar (47.06% vs. 52.94%, *p* value >0.05). Similar accuracy was observed in VASP and APACHE III score in predicting mortality of lung cancer (84.37% vs. 85.77%, *p* value>0.05). This paper concludes that the level of VASP correlates to the severity of the lung cancer and survival of the patients.

## 1. Introduction

Medical check-ups are more common in China due to the increasing reports of environmental issues. The incidence of lung cancer has been on the rise in recent years. Now it is the leading cause of tumor. Despite the continuous progress in the diagnosis and treatment of lung cancer, no significant improvement was achieved in its prognosis and patients' survival time [1–7]. To make matters worse, the prognosis and survival rate of lung cancer noticeably decrease as it moves to more advanced stages [8–10]. As such, it is critical to detect and treat lung cancer in a timely manner. In recent years, although targeted drug therapy and monoclonal antibody immunotherapy for tumors have been clinically applied, the mortality rate of lung cancer remains high in China. According to data released by the World Health Organization, the incidence of lung cancer in China in 2020 was 17.9% with a mortality rate of 23.8%. It has the highest mortality rate among malignant tumors [11].

The article "Clinical Significance of Detection of Peripheral Blood VASP Level in Lung Cancer Patients" was retracted in 2023. Reasons: unreliable results or conclusions; lack of ethics approval or compliance; concerns about the data; concerns about the peer review.

Vasodilator-stimulated phosphoprotein (VASP) is the protein in the cytoskeleton. In recent years, studies have found that VASP is a cancer-promoting molecule [1]. The deletion of VASP can lead to the generation of tumor cells, and its expression level causes transformation of tumor cells [2, 3]. Interestingly, VASP is highly expressed in lung adenocarcinoma tissues. It correlates strongly with tumor differentiation, lymph node metastasis and invasion, and survival and prognosis of patients [4–7]. The inconsistency on the relationship between the VASP level and the occurrence of tumors warrants further research. Taken together, VASP may be an important tumor diagnosis and prognosis molecule. In light of these facts, both novel treatment measures and early diagnosis help to reduce the mortality rate of lung cancer patients. The current markers widely used in the clinical screening or diagnosis of lung squamous cell carcinoma, adenocarcinoma, and small cell carcinoma include carcinoembryonic antigen (CEA), squamous cell carcinoma antigen (SCC), neuron-specific enolase (NSE), carbohydrate antigen 125 (CA125), cytokeratin-19 fragment (CYFRA21-1), and prosecretin-releasing peptide (proGRP) [12]. Unfortunately, despite the sufficient specificity for diagnosis, the sensitivity is not high for any of these markers. False positives occur due to the interference of benign tumors, inflammation, hormones, and other factors [13]. We planned to include 100 lung cancer patients and 50 healthy people in our study. Furthermore, the lung cancer patients were divided into two groups based on the presence of lymph node metastasis. The recurrence of tumor was determined via the peripheral blood VASP levels in lung cancer patients without lymph node metastasis before and after surgery. The VASP levels before and after chemotherapy in the lung cancer patients treated with chemotherapy were compared to facilitate the prognosis and stratified management of lung cancer.

The article "Clinical Significance of Detection of Peripheral Blood VASP Level in Lung Cancer Patients" was retracted in 2023. Reasons: unreliable results or conclusions; lack of ethics approval or compliance; concerns about the data; concerns about the peer review.

## 2. Materials and Methods

### 2.1. Settings

This study was conducted by the Third Hospital of Hebei Medical University Laboratory. The study is from January 2018 and December 2020. The study protocol was approved by the Institutional Review Board of the Third Hospital of Hebei Medical University (2017-12-11) in compliance with the World Medical Association (WMA) Declaration of Helsinki and its subsequent amendments and the Indian Council of Medical Research (ICMR) on human participation ethical guidelines for biomedical research.

### 2.2. Study Design

This study was prospective, observational, open-label, and single-arm.

### 2.3. Inclusion and Exclusion Criteria

Inclusion criteria were as follows: meet the diagnostic criteria of “Diagnostic Criteria for Primary Lung Cancer” [3]; diagnosed with lung cancer by pathological section and cytology; lung cancer cells were found by pleural effusion examination; history of smoking; patients with cough, expectoration, chest tightness, and shortness of breath; symptoms such as blood in the sputum and fever; chest computed tomography scans showed that there was a mass in the lung with irregular edges and burrs, accompanied by symptoms such as obstructive pneumonia and atelectasis. Exclusion criteria were as follows: patients with other tumors; life expectancy was less than 1 year; patients with mental and cognitive impairments.

### 2.4. Methods

Two millilitre of EDTA anticoagulated venous blood was collected from the healthy control group, the lymph node metastasis group, and the non-lymph node metastasis group, respectively. The VASP levels of all samples were measured by flow cytometry. The flow cytometer NAVIOS was provided by Beckman Company of the United States. The plasma VASP level detection reagents, calibrators, and quality control materials were provided by Jiangxi Saiji Biotechnology Co. Ltd.

At the same time, 8 mL of fasting cubital venous blood was drawn from lung cancer patients in the morning. Electrochemiluminescence and enzyme-linked immunosorbent assays were used to determine serum prosecretin-releasing peptide (proGRP), squamous cell carcinoma antigen (SCC), neuron-specific enolase (NSE), and cytokeratin. The level of cytokeratin-19 fragment (CYFRA21-1) was detected using Roche electrochemiluminescence kit and Elecsys2010 electrochemiluminescence analyzer. The kit and analyzer were purchased from Roche.

### 2.5. Outcome Evaluation

All lung cancer patients' condition was assessed by admission assessment, namely, acute physiology and chronic health evaluations III (APACHE III) score evaluation.

The article "Clinical Significance of Detection of Peripheral Blood VASP Level in Lung Cancer Patients" was retracted in 2023. Reasons: unreliable results or conclusions; lack of ethics approval or compliance; concerns about the data; concerns about the peer review.

### 2.6. Statistical Processing

All data analysis was performed using SPSS 25.0 statistical software. The measurement data of the detection indicators were expressed as *X* ± *S*. The comparison between groups was performed by *t*-test. The count data (rates) were compared using the *X*^2^ test. The diagnostic efficacy was mapped by the receiver operating characteristic (ROC) curve. Survival rates were compared using log-rank analysis. The statistical significance level was set at 0.05 (5% level of significance).

## 3. Results

### 3.1. Baseline Data

Ten participants withdrew from the study because they left Hebei. At the end of the study, 100 participants were included in the final analysis. Totally 100 patients (50–88 years old) were included, including 51 males and 49 females, with an average age of 63 ± 12.63 years. They were further assigned into two groups according to the presence of lymph node metastasis. In the lymph node metastasis group (*n* = 53), there were 27 males and 26 females, with an average age of (65.00 ± 11.75) years. In the non-lymph node metastasis group (*n* = 47), there were 23 males and 24 females, with an average age of (62 ± 13.38) years. The control group composed of 50 healthy individuals from our hospital health screening, including 26 males and 24 females, with an average age of (60.00 ± 10.33) years. The gender and age difference in pairwise comparison among these 3 groups is statistically insignificant (with all 3 *p* values >0.05). The APACHE III score of the lymph node metastasis group was higher than that of the non-lymph node metastasis group. The difference was statistically significant (*p* values <0.01) (see Table 1).

### 3.2. VASP Values and APACHE III Score

The VASP values of the three groups were compared. The difference was statistically significant (*p* value <0.01). The value of VASP in the non-lymph node metastasis group was significantly higher than that in the healthy control group. The VASP level in the lymph node metastasis group was significantly higher than that in the non-lymph node metastasis group and the healthy control group (all *p* values <0.05). The APACHE III score of the lymph node metastasis group was higher than that of the non-lymph node metastasis group (*p* values <0.05) (see Table 2).

### 3.3. Receiver Operating Characteristic (ROC) Curve Analysis

Table 3 summarizes the diagnostic efficacy of VASP based on the receiver operating characteristic (ROC) curve analysis. The result is similar to that of SCC, NSE, CYFRA21-1, and proGRP.

In the end, 17 of 100 lung cancer patients died. The difference of plasma VASP levels in the survival group and the death group was statistically significant, with higher level observed in the death group (all *p* values <0.05, Table 4).

The article "Clinical Significance of Detection of Peripheral Blood VASP Level in Lung Cancer Patients" was retracted in 2023. Reasons: unreliable results or conclusions; lack of ethics approval or compliance; concerns about the data; concerns about the peer review.

The plasma VASP level and APACHE III scores for mortality were similar in lung cancer (47.06% vs. 52.94%, *X*^2^ = 2.234, *p* > 0.05). Similar accuracy was observed in VASP and APACHE III score when it comes to mortality risk (84.37% vs. 85.77%, *X*^2^ = 3.494,*p* value >0.05). This implies that that both indicators could be used to assess the risk of death.

## 4. Discussion

To date, the etiology of lung cancer remains controversial. It was reported 20 years ago that the deletion of VASP can lead to the generation of tumor cells. Its expression level caused transformation of tumor cells. Wang et al. showed that VASP was highly expressed in lung adenocarcinoma tissue [14] and was related to the extent of tumor differentiation. Therefore, VASP may be an important tumor diagnostic and prognostic molecule [15]. However, the clinical significance of VASP in lung squamous cell carcinoma is yet to be fully understood. VASP was originally found in platelets as a cytoskeletal protein that regulates intercellular adhesion, cell motility, and morphological changes [16].

In recent years, relevant studies have shown that VASP may be a cancer-promoting factor. It was found that VASP is expressed in breast cancer patients. Artificial overexpression of VASP in *in vitro* experiments promotes the migration and invasion of breast cancer cells [17]. The mechanism is assumed to be inducing epithelial-mesenchymal transition in breast cancer cells. Pang reported highly expressed VASP genes in lung squamous cell carcinoma [18]. Such expression was also closely related to lymph node metastasis and unfavorable clinical prognosis in lung cancer patients. VASP was an independent prognostic factor for lung squamous cell carcinoma. Its expression level is of considerable clinical significance for the prognosis of lung cancer in patients. Similarly, Zhang et al. and Tu et al. obtained the same conclusion in gastric and colon cancer, respectively [19]. However, there is a paucity of report regarding the evidence of the correlation between the level of VASP in peripheral blood, the pathogenesis, and the severity of lung cancer.

Our results show that the level of plasma VASP in the healthy control group is statistically lower than that in lymph node metastasis group, which is in turn statistically lower than that in non-lymph node metastasis group. The APACHE III score is found to increase with the aggravation of lung cancer, suggesting that VASP has a positive correlation with the presence and the severity of lung cancer. Multivariate regression analysis shows that the efficacy of plasma VASP level in diagnosing lung cancer is similar to that of SCC, NSE, CYFRA21-1, and proGRP. It is suggested that the plasma VASP level can be adopted in early diagnosis of lung cancer. Moreover, the plasma VASP level in the death group was higher than that in the survival group. The plasma VASP level for lung cancer mortality is comparable to that of SCC, NSE, CYFRA21-1, and proGRP. At present, the APACHE III score is used clinically to assess the condition of critically ill patients and to evaluate the prognosis [20]. Higher score correlates with more severe condition, worse prognosis, and higher mortality. Additionally, our study shows that plasma VASP has a similar accuracy to APACHE III in predicting the lung cancer mortality risk. This indicates that the risk of death of lung cancer can be assessed by the plasma VASP levels.

The article "Clinical Significance of Detection of Peripheral Blood VASP Level in Lung Cancer Patients" was retracted in 2023. Reasons: unreliable results or conclusions; lack of ethics approval or compliance; concerns about the data; concerns about the peer review.

In view of the low sensitivity of many diagnostic methods, the possibility of false positives, and the fact that the use of VASP is still in the experimental stage, a Chinese medicine “Zhongtu theory” explores the traditional Chinese medicine (TCM) treatment of lung cancer [18] and its impact on the function of various organs. Disorders and the formation of pathological products are closely related to spleen-earth dysfunction. The “phlegm” and “drinking” in lung cancer are prominent. “Phlegm” and “drinking” are not only the pathological products of lung cancer but also the aggravating factors of the disease. Moreover, with the progress of lung cancer, phlegm-drinking increases day by day. Damp phlegm accumulates and occludes the lung, causing difficulty in breathing. This problem is more prominent in advanced-stage patients, who suffer from pleural and pericardial effusion, which is the cohesion of phlegm-drinking. Therefore, it can be used as a differential diagnosis for clinical features at this time. If this feature occurs, patients ought to seek medical attention in time to avoid further delays. The high expression of hypoxia-inducible factor 1a and vascular endothelial growth factor in lung cancer cells alongside “phlegm” and “drinking” promotes tumor angiogenesis. At the same time, it stimulates matrix metalloproteinase-2 and urokinase-type plasminogen activator, resulting in lung cancer cell invasion. Therefore, taken together the molecular and the TCM point of view, patients should seek medical treatment in time when experiencing clinical symptoms. The VASP sequence consists of 380 amino acids, of which 3 are phosphorylation sites, 2 are serine sites (Ser157 and Ser 239), and the other is a threonine site (Thr 278). The three phosphorylation sites directly receive protein kinase k and protein kinase A regulation, and VASP phosphorylation is closely related to its function. Based on network pharmacology “drug-target-disease,” Aidi injection can regulate VASP phosphorylation and reduce its expression. Aidi injection mainly consists of cantharidin, ginseng, astragalus, and Acanthopanax senticosus, and the auxiliary material is glycerol (for injection) [21], which can enhance the body's non-specific and specific immune function and improve the body's ability to stress. The combination of cancer drugs 5-Fu and CTX and the concurrent treatment with radiotherapy have synergistic effects, which can keep leukocytes and platelets in the normal range and reduce the expression of VASP. In vitro experiments show that Aidi injection can directly kill and inhibit cancer cells.

The article "Clinical Significance of Detection of Peripheral Blood VASP Level in Lung Cancer Patients" was retracted in 2023. Reasons: unreliable results or conclusions; lack of ethics approval or compliance; concerns about the data; concerns about the peer review.

## 5. Conclusion

The expression of VASP in tumor tissue is highly related to cancer cell invasion, metastasis, prognosis, and survival rates in patients. The expression of VASP in gastric cancer [22] is positively correlated with its pathological grade, which is also similar to the results of this study that the level of VASP is related to the severity of lung cancer and the survival rate of patients. These findings would suggest that VASP is involved in the differentiation of normal gastric mucosal epithelial cells into cancer cells and VASP is an important molecule regulating the invasive properties of gastric cancer. Additionally, VASP is involved in regulating the invasion ability of prostate cancer PC3 cells [23], and the difference of VASP expression is related to the prognosis of prostate cancer patients. As indicated, VASP is used as a predictor of disease progression or survival time in cancer patients, but it has not been deeply explored in this study and it will be included in the research plan in the future. Firstly, VASP genes are highly expressed in lung cancer cells. It is thus closely related to lymph node metastasis and poor prognosis of lung cancer. The reduction of VASP level inhibits the metastasis of lung cancer cells in vitro. It can thus serve as a molecular indicator in diagnosis and treatment [21]. The plasma VASP level in patients with lung cancer is higher than that in the control group. The VASP level in the patients without lymphocyte metastasis is higher than that in the lymphocyte metastasis group. Secondly, the increase of its level might reflect the severity of the disease. The mortality risk in patients with higher level of VASP is higher. This indicates that VASP is possibly involved in the development and prognosis of lung cancer. Thirdly, its correlation with the severity of lung cancer aids in early diagnosis and treatment of lung cancer. This further reduces the mortality rate of lung cancer patients. In conclusion, measuring the VASP level in lung cancer patients allows us to better evaluate their conditions and prescribe treatments.

The article "Clinical Significance of Detection of Peripheral Blood VASP Level in Lung Cancer Patients" was retracted in 2023. Reasons: unreliable results or conclusions; lack of ethics approval or compliance; concerns about the data; concerns about the peer review.

By reasonable guesses, the treatment and prognosis of VASP are different from existing treatments. This may be due to the small number of patients included and the lack of multicenter studies, which might bias the results.

## Figures and Tables

**Table 1:** Comparison of baseline features of healthy control group, non-lymph node metastasis group, and lymph node metastasis group.

Groups	*n*	Gender		Age (year, *x* ± *s*)	APACHE III score (*x* ± *s*)
		Male	Female		
Healthy control group	50	26	24	60 ± 10.33	—
Non-lymph node metastasis group	47	23	24	62 ± 13.38	12.4 ± 3.9
Lymph node metastasis group	53	27	26	65 ± 11.75	19.97 ± 3.82
*X* ^2^/*F*/*t*		1.342	3.439	4.231	
*p*		0.231	0.323	<0.01	

**Table 2:** Plasma VASP levels and APACHE III score.

Groups	*n*	VASP (pg/ml)	APACHE III score (point, *x* ± *s*)
Healthy control group	50	2.05 ± 1.24	—
Non-lymph node metastasis group	47	15.22 ± 3.14^*a*^	12.4 ± 3.9
Lymph node metastasis group	53	39.59 ± 6.43^*ab*^	19.97 ± 3.82
*F*/*t*		2.763	4.421
*p*		<0.01	<0.01

*Note.* Compared with the healthy control group, ^*a*^*p* < 0.05; compared with the non-lymph node metastasis group, ^*b*^*p* < 0.05.

**Table 3:** Comparison of diagnostic efficacy between VASP and SCC, NSE, CYFRA21-1, and proGRP.

	AUC	Standard error	Sig	95% CI
SCC	0.891	0.023	0.000	0.839–0.942
NSE	0.887	0.033	0.000	0.778–0.891
CYFRA21-1	0.885	0.028	0.000	0.835–0.939
proGRP	0.897	0.038	0.000	0.842–0.945
VASP	0.873	0.029	0.000	0.836–0.979

**Table 4:** VASP levels in survival and death groups (*X* ± *S*).

Groups	*n*	VASP (pg/ml)	SCC (pg/ml)	NSE (pg/ml)	CYFRA21-1 (pg/ml)	proGRP (pg/ml)
Survival group	83	22.33 ± 4.75	32.14 ± 9.98	49.38 ± 12.15	30.22 ± 9.25	58.26 ± 11.76
Death group	17	53.22 ± 2.01	81.62 ± 20.58	162.85 ± 36.19	92.43 ± 23.52	123.45 ± 35.69
*T*		1.324	1.532	2.432	1.834	3.231
*p*		0.01	<0.01	<0.01	<0.01	<0.01

## Data Availability

The data generated or analyzed during this study are included within the article.
